The article "LINC00675 is a prognostic factor and regulates cell proliferation, migration and invasion in glioma" was published in 2018. Journal: Biosci Rep.

# LINC00675 is a prognostic factor and regulates cell proliferation, migration and invasion in glioma

**DOI:** 10.1042/BSR20181039

**Published:** 2018-09-19

**Authors:** Zhibing Li, Yijian Li, Qibai Wang

**Affiliations:** 1 Department of Neurology, Shanxi Provincial Tumor Hospital, Taiyuan 030003, Shanxi, China; 2 Second Department of Surgery, Traditional Chinese Medicine Hospital of Juye County, Heze 274900, Shandong, China; 3 Department of Neurology, Hospital of Chongqing Red Cross Society, Jiangbei District People’s Hospital, Chongqing 400025, China

**Keywords:** biomarkers, cancer, glioma, LINC00675, large intervening non-coding RNA, prognosis

## Abstract

LINC00675 has been suggested to be dysregulated in gastric cancer, colorectal cancer and pancreatic cancer. However, the expression status and biological function of LINC00675 in glioma were still unknown. Thus, we reported LINC00675 was overexpressed in glioma tissues and cell lines, and positively associated with advanced WHO grade, large tumor size and poor prognosis. Moreover, univariate and multivariate analyses suggested that high-expression of LINC00675 was an independent unfavorable prognostic predictor for glioma. In addition, levels of LINC00675 expression were positively correlated with TRIP6 mRNA and protein expressions. The *in vitro* experiment showed that silencing of LINC00675 inhibits glioma cell proliferation, migration and invasion through regulating TRIP6. In conclusion, LINC00675 acts as a tumor promoter in glioma progression.

## Introduction

Glioma originates in the glial cells and is the most common primary central nervous system malignant tumor [1]. The gliomas were divided into World Health Organization (WHO) grades I–IV based on increasing levels of malignancy, such as well-differentiated low-grade astrocytomas (WHO grade I-II), anaplastic astrocytomas (WHO grade III) and glioblastoma multiforme (WHO grade IV) [2]. An upward trend in morbidity and mortality for glioma observed from 2000 to 2011 in China [3,4]. According to Cancer Statistics in China, glioma is the seventh common cancer in China, with an estimated 101,600 new cases and 61,000 deaths in 2015 [3]. Although the treatment strategies of surgical resection, radiation and chemotherapy for glioma patients have been greatly improved, the overall survival time remains dissatisfactory, especially for high-grade glioma [5–7]. Therefore, it is urgent to elucidate molecular mechanisms of glioma tumorigenesis for developing novel treatments for gliomas.

Long non-coding RNAs (LncRNAs) is a wide variety of RNA transcripts of sizes greater than 200 nucleotides (nt) that lack significant protein-coding capacity [8]. Recently, several lncRNAs have been suggested to as key elements of glioma tumorigenesis, such as DANCR [9,10], PVT1 [11], SNHG6 [12], XIST [13], HOTTIP [14], H19 [15], HULC [16] and so on.

LINC00675 (also known as TMEM238L) has been shown to be dysregulated and as a prognostic predictor in gastric cancer [17], colorectal cancer [18] and pancreatic cancer [19]. The expression status and prognostic value of LINC00675 in glioma are still unknown. In order to explore the role of LINC00675 in glioma, we analyze TCGA (The Cancer Genome Atlas) database that includes 641 glioma cases and found glioma patients with high-expression of LINC00675 had shorter disease-free survival and overall survival time than those with low-expression of LINC00675. Then, we guess that LINC00675 serves as an oncogenic lncRNA in glioma. Therefore, the purpose of our study is to investigate the clinical significance in clinical samples and biological function of LINC00675 in glioma cells.

## Materials and methods

### TCGA database analysis

Transcriptional abundance of glioma-related LINC00675 was excavated from The Cancer genome Atlas (TCGA, http://cancergenome.nih.gov). In brief, a total of 641 glioma specimens were available for the survival analysis.

### Patient tissue specimens

Fresh 118 tumor tissue specimens and 15 paired peritumoral tissue specimens from 118 glioma patients, who underwent radical tumor resection at Shanxi Provincial Tumor Hospital and Hospital of Chongqing Red Cross Society, were enrolled for qRT-PCR. None of the patients had received radiotherapy or chemotherapy prior to surgery. Based on the 2007 edition of World Health Organization (WHO) central nervous system tumor grading criteria, all cases were divided into I–IV level. The present study was approved by the Ethics Committee of Shanxi Provincial Tumor Hospital and Hospital of Chongqing Red Cross Society, and written informed consent was obtained from all the patients.

### RNA isolation and qRT-PCR

RNA was extracted from tissues and cells using Trizol (Takara, Japan) per the manufacturer’s protocol. The cDNA was synthesized from 1 μg of total RNA with PrimeScript^®^ RT reagent Kit (Takara, Japan). Real-time PCR was performed with the SYBR^®^ Premix Ex TaqTM II (Takara, Japan) detection method on an ABI-7500 RT-PCR system. The β-actin gene was used as gene internal control. All the primers were listed as follows: LINC00675 forward, 5′-GCCTACTG CTCTGGATCATCTGGTA-3′; reverse, 5′-ACCTGCG TCTCTTCTCCTCTTCC-3′. β-actin forward, 5′-TTCCTTCCTGGGCATGGAGTCC-3′; reverse, 5′-TGGCGTACAGGTCTTTGCGG-3′.

### Cell culture

The human glioma cell lines (Hs683, U251, U-87 and A-172) and a normal brain glial cell line (HEB) were purchased from the Chinese Academy of Sciences (Shanghai, China) and maintained in Dulbecco’s Modified Eagle Medium (DMEM, Hyclone, U.S.A.) containing 10% fetal bovine serum (FBS, GIBCO, U.S.A.). All cell lines were cultured at 37°C in a humidified atmosphere of 5% CO_2_.

### Cell transfection

The siRNAs targeting LINC00675 and the corresponding negative control were synthesized by GenePharma Company (Suzhou, China). Three siRNAs were designed to silence LINC00675 expression. The target site one (si-LINC00675) is the most effective site and is chosen for further study. Cell transfection was performed with lipofectamine 3000 (Invitrogen, U.S.A.), according to the manufacturer’s instructions.

### MTT analysis

LINC00675-silenced U-87 and A-172 cells were seeded at a density of 1000 cells per well in 96-well plates. After 1, 2, 3 or 4 days, cell viability was analyzed using MTT (3-(4, 5-dimethylthiazol-ayl)-2, 5-diphenyl tetrazolium bromide) assay. At the indicated time points, 10 μl of 5 mg/ml MTT was added to each well, and cells were incubated for 4 h at 37 °C. The media was then discarded, and 150 μl of DMSO was added to each well for 20 min. The optical density (OD) was detected at 490 nm with a microplate reader. All assays were independently repeated three times.

### Cell cycle analysis

Cells were harvested and washed with phosphate buffer saline (PBS), then fixed in 70% ice-cold ethanol overnight. The fixed cells were incubated with PBS containing 10 μg/ml propidium iodide and 0.5 mg/ml RNase A for 15 min at 37°C. The FC500 flow cytometry system (Beckman Coulter, U.S.A.) was used to gain the DNA content of labeled cells. All assays were independently repeated three times.

### Cell migration and invasion assays

LINC00675-silenced U-87 and A-172 cells were diluted to a density of 2.5 × 10^5^ per ml. Next, 200 μl of the cells were added into a transwell chamber (Costar, U.S.A.) without or with Matrigel (BD, U.S.A.). After 24 h, the chamber was stained with Giemsa solution, and the cells in the inside of the chamber were wiped off. Then, the cells on the outside of the chamber were counted in under a microscope in five predetermined fields. All assays were independently repeated three times.

### Western blot

Total protein was extracted from cells using RIPA protein extraction reagent (Beyotime, China) and was quantified using the BCA protein assay kit (Beyotime, China). Equal amounts (50 μg) of protein was separated by 10% SDS-PAGE and transferred on PVDF membrane. The target proteins were incubated with the following primary antibodies: TRIP6 antibody (dilution: 1:1000, Abcam, U.S.A.) or β-actin antibody (dilution: 1:3000, CWBIO, China). Signals were detected using enhanced chemiluminescence reagents (Pierce, U.S.A.) and analyzed by Quantity One Software (Bio-Rad, U.S.A.).

### Immunohistochemical staining

Thirty paraffin-embedded glioma sections were used for immunohistochemistry to detect protein expression levels of TRIP6 through TRIP6 antibody (dilution: 1:200, Abcam, U.S.A.). The indirect streptavidin-peroxidase method was utilized based on the manufacturer’s instructions. Stained tissue sections were reviewed and scored separately by two pathologists blinded to the clinical parameters. Any disagreements were arbitrated by the third pathologists. The staining intensity was scored as previously described [20]. Briefly, the intensity of immunostaining was 0–3 (negative: 0; weak: 1; moderate: 2; strong: 3), and staining extent was scored as (0–25%): 1, (26–50%): 2, (51–75%): 3 and (76–100%): 4. The final score was calculated by multiplication of intensity and extent score. Low-expression of TRIP6 was defined as 0–4 scores; high-expression of TRIP6 was defined as more than 4 scores.

### Statistical analysis

Statistical analyses were performed using SPSS 17.0 (SPSS Inc., Chicago, U.S.A.). Differences among groups in *in vitro* studies were analyzed for statistical significance by two-tailed unpaired Student’s independent samples *t* tests. The Wilcoxon Signed Rank test was conducted to compare the expression of LINC00675 between glioma tissues and paired peritumoral tissues. The chi-square test was used to investigate the association between LINC00675 expression and clinicopathological parameters of glioma patient. Differences of survival times between LINC00675 high-expression group and LINC00675 low-expression group were detected using the Kaplan and Meier survival curves, and compared by the log-rank test. The prognostic significance of various variables was analyzed by univariate and multivariate survival analysis using Cox’s regression model. The relationship between LINC00675 expression and TRIP6 mRNA level was detected by using Spearman’s correlation coefficient analysis. *P* value <0.05 was considered statistically significant.

## Results

### Levels of LINC00675 expression are increased in glioma tissues and cell lines

In order to explore the expression of LINC00675 in glioma, we analyzed LINC00675 expression in glioma tissues, paired peritumoral normal tissues, glioma cell lines and normal brain glial cell line. LINC00675 suggested a significantly higher expression level in glioma tissues compared with peritumoral normal tissues (*P*<0.001, Figure 1A). Compared with normal brain glial cell line (HEB), LINC00675 levels were notably increased in glioma cell lines (Hs683, U251, U-87 and A-172) (*P*<0.001, Figure 1B). Interestingly, we observed that LINC00675 expression was higher in high-grade glioma cell lines (U-87 and A-172) than in low-grade glioma cell lines (Hs683 and U251) (*P*<0.001, Figure 1B). This suggests that LINC00675 expression may associated with aggressive status of glioma cell.

**Figure 1:** Levels of LINC00675 expression are increased in glioma tissues and cell lines (**A**) The expression of LINC00675 is detected in 15 pairs of glioma tissues and peritumoral normal tissues. (**B**) The expression of LINC00675 is measured in glioma cell lines (Hs683, U251, U-87 and A-172) and normal brain glial cell line (HEB). (**C**) The efficiency of si-LINC00675 is confirmed by qRT-PCR in U-87 and A-172 cells.

### LINC00675 high-expression associated with the malignant status of glioma cases

We detected LINC00675 expression in 118 glioma samples through qRT-PCR and investigated the correlation between LINC00675 expression and clinicopathological variables of glioma patients. Based on published study [21], we divided all glioma cases into two groups according to LINC00675 expression: LINC00675 high-expression group (*n*=59) and LINC00675 low-expression group (*n*=59). As summarized in Table 1, high-expression of LINC00675 was dramatically associated with advanced WHO grade (I–II vs. III–IV; *P*=0.007) and large tumor size (<3 cm vs. ≥3 cm, *P*=0.008). However, LINC00675 expression was not correlated with age (*P*=0.343), gender (*P*=0.196), family history of cancers (*P*=0.665) and tumor location (*P*=0.170).

**Table 1:** Correlations between LINC00675 expression and clinicopathological characteristics in glioma

Characteristics	*n*	High expression (%)	Low expression (%)	*P*
Age (years)				
<45	45	25(55.6)	20(44.4)	0.343
≥45	73	34(46.6)	39(53.4)	
Gender				
Male	63	28(44.4)	35(55.6)	0.196
Female	55	31(56.4)	24(43.6)	
Family history of cancer				
Yes	28	13(46.4)	15(53.6)	0.665
No	90	46(51.1)	44(48.9)	
WHO grade				
I-II	42	14(33.3)	28(66.7)	0.007
III-IV	76	45(59.2)	31(40.8)	
Tumor size (cm)				
<3	46	16(34.8)	30(65.2)	0.008
≥3	72	43(59.7)	29(40.3)	
Tumor location				
Supratentorial	94	44(46.8)	50(53.2)	0.170
Infratentorial	24	15(62.5)	9(37.5)	

### LINC00675 high-expression predicts a poor prognosis in glioma patients

In order to explore the prognostic value of LINC00675 in glioma patients, we analyzed a cohort included 641 glioma cases from TCGA database. We found glioma patients with high-expression of LINC00675 had shorter disease-free survival (*P*<0.001, Figure 2A) and overall survival time (*P*<0.001, Figure 2B) than those with low-expression of LINC00675. Similarly, our study showed that levels of LINC00675 were negatively correlated with the overall survival of glioma cases (*P*<0.001, Figure 2C). Furthermore, Univariate and multivariate Cox proportional hazard models were used to analyze the value of various clinical parameters in survival. The univariate analyses suggested that WHO grade, tumor size and LINC00675 expression were markedly correlated with overall survival of glioma patients (*P*<0.001, *P*=0.005 and *P*<0.001, respectively; Table 2). Then, multivariate analyses indicated that high-expression of LINC00675 was an independent unfavorable prognostic predictor for glioma (HR, 95%CI: 2.110, 1.248–3.569; *P*=0.005; Figure 1C).

**Figure 2:** LINC00675 overexpression predicts a poor prognosis in glioma patients (**A**) Increased LINC00675 levels are correlated with short disease-free survival of glioma patients from TCGA database. (**B**) Increased LINC00675 levels are correlated with short overall survival of glioma patients from TCGA database. (**C**) Increased LINC00675 levels are correlated with short overall survival of Chinese glioma patients from our study.

**Table 2:** Univariate and multivariate Cox regression analyses of overall survival

Parameter	Univariate analysis			Multivariate analysis		
	HR	95%CI	*P*	HR	95%CI	*P*
Age (years)						
(<50 vs. ≥50)	1.066	0.650–1.748	0.800			
Gender						
(male vs. female)	1.279	0.786–2.080	0.322			
Family history of cancer						
(yes vs. no)	0751	0.432–1.307	0.311			
WHO grade						
(I-II vs. III-IV)	5.782	3.079–10.859	<0.001	4.597	2.324-9.096	<0.001
Tumor size (cm)						
(<3 vs. ≥3)	2.148	1.253–3.682	0.005	1.079	0.595-1.957	0.801
Tumor location						
(supratentorial vs. infratentorial)	1.757	0.968–3.189	0.064			
LINC00675						
(low vs. high)	2.863	1.716–4.775	<0.001	2.110	1.248-3.569	0.005

Abbreviations: 95% CI, 95% confidence interval; HR, hazard ratio.

### Silencing of LINC00675 inhibits glioma cell proliferation, migration and invasion

In order to investigate the effect of LINC00675 on glioma cell viability, migration and invasion, we conducted loss-of-function studies through si-LINC00675 in U87 and A-172 cells. The transfection efficiency of si-LINC00675 was confirmed by qRT-PCR in U87 and A-172 cells (Figure 1C). The results of MTT assay indicated that silencing of LINC00675 markedly depressed glioma cell viability compared with the control groups (*P*<0.05, Figure 3A). Moreover, cell cycle analyses suggested that silencing of LINC00675 strikingly inhibited cell cycle progression from G1 to S phase (*P*<0.05, Figure 3B). The results of cell migration assay showed the migrated cells in si-LINC00675 groups was notably less than the si-control groups (*P*<0.001, Figure 3C). Consistent with cell migration assays mentioned above, the invasion assay indicated that si-LINC00675 groups had decreased invasive ability compared with than si-control groups (*P*<0.001, Figure 3D).

**Figure 3:** Silencing of LINC00675 inhibits glioma cell proliferation, migration and invasion (**A**) Silencing of LINC00675 depresses cell proliferation in U-87 and A-172. (**B**) Silencing of LINC00675 blocks cell cycle progression from G1 to S phase. (**C**) Silencing of LINC00675 inhibits cell migration in U-87 and A-172. (**D**) Silencing of LINC00675 represses cell invasion in U-87 and A-172. *P<0.05; **P<0.001 .

### LINC00675 positively regulates TRIP6 expression in glioma

TRIP6 has been suggested to be dysregulated in multiple cancers and plays pleiotropic roles in tumor initiation, tumor growth and metastasis [22]. To investigate the molecular mechanism of LINC00675 involved in glioma tumorigenesis, we observed LINC00675 expression was significantly positively associated with TRIP6 expression in glioma from TCGA database (*r*=0.552, *P*<0.001, Figure 4A). Furthermore, the association of LINC00675 expression with TRIP6 mRNA and protein was further investigated in glioma tissue samples. We observed that levels of LINC00675 expression were positively correlated with TRIP6 mRNA expression (*r*=0.654, *P*=0.008, Figure 4B) and TRIP6 protein expression (*r*=0.566, *P*=0.001, Figure 4C and Table 3). Then, we observed that silencing of LINC00675 dramatically inhibited TRIP6 mRNA and protein expressions in U87 and A-172 cells (Figure 3D,E).

**Figure 4:** LINC00675 positively regulated TRIP6 expression in glioma (**A**) LINC00675 expression is significantly positively associated with TRIP6 expression in glioma from TCGA database. (**B**) LINC00675 expression is significantly positively associated with TRIP6 expression in glioma from our study. (**C**) Immunohistochemical staining of TRIP6 in glioma: (a) negative expression in low-grade glioma; (b) low expression in low-grade glioma; (c) high-expression in low-grade glioma; (d) negative expression in high-grade glioma; (e) low expression in high-grade glioma; (f) high-expression in high-grade glioma. (**D**) Silencing of LINC00675 inhibits TRIP6 mRNA expression in U87 and A-172. (**E**) Silencing of LINC00675 represses TRIP6 protein expression in U87 and A-172.

**Table 3:** The association between LINC00675 and TRIP6 protein in glioma

Group		*n*	TRIP6 protein		*R*	*P*
			High expression	Low expression		
Linc00675	High expression	15	14	1	0.566	0.001
	Low expression	15	6	9		

## Discussion

LINC00675 is located in the human chromosome 17p13.1-p12 and has been found to be dysregulated in various human cancers. Originally, Li et al. [19] analyzed a microarray targeting 7419 lncRNAs and found that LINC00675 in pancreatic cancer tissues was 672 times that in chronic pancreatitis tissue. Furthermore, the high-expression LINC00675 was confirmed through qRT-PCR in pancreatic ductal adenocarcinoma tissues and cell lines compared with matched adjacent non-tumor tissues and human pancreatic ductal epithelial cell line, respectively [19]. Subsequently, Zeng et al. [17] conducted lncRNA microarray including five pairs of gastric cancer and the adjacent normal tissues and found that LINC00675 was down-regulated in gastric cancer tissues compared with adjacent normal tissues. The level of LINC00675 was further confirmed in gastric cancer tissues, adjacent non-tumor tissues and healthy gastric mucosa tissues, and found that levels of LINC00675 were reduced in gastric cancer tissues compared with adjacent non-tumor tissues or healthy gastric mucosa tissues. Similarly, Shan et al. [18] reported that the expression of Linc00675 was decreased in colorectal cancer tissues and cells. However, the expression status and prognostic value of LINC00675 in glioma were still unknown. We analyzed LINC00675 expression in glioma tissues, paired peritumoral normal tissues, glioma cell lines and normal brain glial cell line, and found that LINC00675 levels were notably increased glioma tissues and cell lines compared with peritumoral normal tissues and normal brain glial cell line, respectively. Moreover, we further investigated the correlation between LINC00675 expression and clinicopathological variables of glioma patients, and found the high-expression of LINC00675 was dramatically associated with advanced WHO grade and large tumor size. Similarly, Li et al. [19] showed that LINC00675 overexpression positively associated with lymph node metastasis and perineural invasion. Contrarily, Shan et al. indicated that LINC00675 low expression was markedly correlated with advanced clinical stage, present lymph node metastasis and high level of CEA [17]. Meanwhile, Shan et al. [18] revealed that LINC00675 expression was also relatively low in metastatic colorectal cancer tissues and advanced colorectal cancer tissues. Together, these data suggested that the expression status and clinical value of LINC00675 may be different in different types of cancers.

Recently, the prognostic significance of LINC00675 has been reported in gastric cancer [17] and pancreatic cancer [19]. In gastric cancer patients, a worse overall survival rate was observed in patients with low expression of LINC00675 [17]. Oppositely, LINC00675 high-expression was positively associated with poor overall survival and served as an independent poor prognostic factor in pancreatic cancer patients [19]. In order to the prognostic value of LINC00675 in glioma patients, we analyzed a cohort included 641 glioma cases from TCGA database, and found that patients with high-expression of LINC00675 had shorter disease-free survival and overall survival time than those with low expression of LINC00675. Furthermore, we explore the association between LINC00675 and overall survival in Chinese glioma patients from our study, and found that levels of LINC00675 were negatively correlated with the overall survival of glioma cases. In addition, univariate and multivariate analyses suggested that high-expression of LINC00675 was an independent unfavorable prognostic predictor for glioma.

The biological function of LINC00675 in cancer cells may depend on the specific cancer types. In gastric cancer, LINC00675 overexpression inhibited cell proliferation, migration and invasion *in vitro* and also suppressed the growth and metastases of gastric cancer cells *in vivo* [17]. Moreover, Shan et al. [18] demonstrated that overexpression of LINC00675 depresses colorectal cancer cell proliferation, invasion and migration *in vitro*. However, LINC00675 suppression inhibited pancreatic cancer cell proliferation, invasion and the process of epithelial mesenchymal transition [19]. In our study, we found silencing of LINC00675 markedly depressed glioma cell viability, migration, invasion and cell cycle progression from G1 to S phase. Thus, LINC00675 functioned as tumor promoter in glioma.

In order to investigate the molecular mechanism of LINC00675 involved in glioma tumorigenesis, we observed LINC00675 expression was significantly positively associated with TRIP6 expression in glioma from TCGA database. TRIP6 has been suggested to be dysregulated in multiple cancers and plays pleiotropic roles in tumor initiation, tumor growth and metastasis [23–26]. In glioma, TRIP6 was overexpressed in all types of gliomas and negatively associated with poor clinical outcomes [27]. Lai et al. [28] reported that TRIP6 high-expression has a notable impact on induced NF-κB activity, resistance to apoptosis and Fas-mediated cell invasion in glioma. Thus, we further investigated the association of LINC00675 expression with TRIP6 mRNA and protein in glioma tissues and cells, and found that levels of LINC00675 expression were positively correlated with TRIP6 mRNA and protein expressions, and silencing of LINC00675 dramatically inhibited TRIP6 mRNA and protein expressions in glioma cell. Thus, LINC00675 might modulate TRIP6 to regulate glioma cell proliferation, migration and invasion.

In conclusion, LINC00675 is overexpressed in glioma tissues and cell lines and positively associated with advanced WHO grade, large tumor size and poor prognosis. Silencing of LINC00675 inhibits glioma cell proliferation, migration and invasion through regulating TRIP6.

## Abbreviations

95% CI: 95% confidence interval
HR: hazard ratio
LncRNA: long non-coding RNA
NF-κB: nuclear factor-kappa B
qRT-PCR: quantitative real-time polymerase chain reaction
